# Study on the Application of Visual Communication Design in APP Interface Design in the Context of Deep Learning

**DOI:** 10.1155/2022/9262676

**Published:** 2022-06-20

**Authors:** Hui Luo, Qiang Zeng

**Affiliations:** ^1^School of Art and Design, Shaoyang University, Shaoyang, Hunan, China; ^2^College of Arts, Huzhou University, Huzhou, Zhejiang, China

## Abstract

Visual communication concepts enable linguistics or semiotics to the teaching of visual communication designs, creating graphic designs into an innovative and scientific discipline. The use of storyline techniques in visual communication not only inspires the imagination of designer but also arouses the visual memory of the audience. Besides, improving cultural heritage such as historical images is important to protect cultural diversity. Recently, the developments of deep learning (DL) and computer vision (CV) approaches make it possible for the automatic colorization of grayscale images into color images. Also, the usage of visual communication design in APP interface design has increased. With this motivation, this work introduces the enhanced deep learning-based automated historical image colorization (EDL-AHIC) technique for wireless network-enabled visual communication. The proposed EDL-AHIC technique intends to effectually convert the grayscale images into color images. The presented EDL-AHIC technique extracts the local as well as global features. For global feature extraction, the enhanced capsule network (ECN) model is applied. Finally, the fusion layer and decoding unit are employed to determine the output, i.e., chrominance component of the input image. A comprehensive experimental validation process is performed to ensure the betterment of the EDL-AHIC technique. The comparison study reported the supremacy of the EDL-AHIC technique over the other recent methods.

## 1. Introduction

It is impossible to develop visual communication without the use of colors and pictures, since they have a significant influence on our perception of the world. The three primary components of a visual media design are color, graphics, and text [1]. When it comes to creating optical media, people will not disregard the importance of color. The goal of visual communication design is to increase the number of people who see and appreciate a company's products by enhancing their visual appeal and creativity. Even though AI technology in multimedia has only been around for a short time, it has already made significant strides, as seen by the emergence of multimedia players and smart voice speakers. Similar to the design of visual media communication, artificial intelligence technology may be used to create a more visual style and a better creative outcome when applied to visual media [2]. For example, cross-media platform dynamic design incorporates several graphic components. Adapting to the current development trends and popular aesthetic desires, these features are becoming more and more prevalent [3]. In a static form, the three components may convey sensory pleasure and psychological resonance to the audience. The dots, lines, and levels of various forms in extended drawings are beneficial for increasing the contrast with the sketch's look, and the text is important for showing the specifics of the images accurately and immediately [4]. Because of the M-shaped socioeconomic structure, consumers now have access to a whole new way of thinking about fashion. Modern customers are used to browsing and purchasing apparel and information swiftly and easily because of the widespread use of Internet connectivity and portable mobile devices [5]. Formal studies may be conducted using simulated websites and surveys to examine product photographs that integrate three visual codes (product, character, and surroundings) and see which of them can generate psychological simulations [6]. People, on the other hand, continue to use antiquated visual communication strategies. Visual communication design and communication science are elements of the equation. Visual communication design's symbols, on the other hand, are difficult to put into words [7]. This is why it is difficult for the audience to accept and comprehend. As a result, designers integrate communication theory into their work and provide a solid theoretical foundation for visual communication design. Using this method, data may be efficiently sent, opening a new avenue for visual communication design study [8]. Nevertheless, this research hypothesis did not substantially stimulate the growth and innovation of visual communication design. Next-generation AI and blockchain technologies are described as providing new ideas for accelerating biomedical research and empowering patients with new tools for controlling their personal data, as well as providing incentives for continuing health monitoring [9]. Data combinations, time, and connection values are some of the new ideas that they created to help people assess and evaluate their own records. Their study data, however, are yet to be verified. The artificial technology plays a greater role in computer vision and APP interface design as well. This study focused on evaluating the application of visual communication in APP interface design using the deep learning technique.

## 2. Related Studies

The design of information transmission via the use of visual symbols is known as “visual communication [10].” Many new technologies have emerged as a result of advancements in science. These include not just printing art but also graphics, electronics, and multimedia design. This information must be “sent” to the audience in order for visual communication to be successful [11]. When it comes to communication design, the goal is to make the other person comprehend. The term “visual symbol” refers to a wide range of media, including photographs, television, movies, video games, and other design items, as well as scientific and literary writings and articles [12]. These four steps address who, what, when, and with whom you should communicate.

The following are some of the most important aspects of visual media color design:

1. Color and image are inextricably related in visual media communication design. In addition to reflecting the thing and its existence, a design must also be original and attractive.
2. There is a strong connection between the text and the color. As a result, the writing has a distinct tone, whether religious or political. Because of this, the symbolism of color must be taken into account while designing the text's color scheme.
3. A variety of things must be taken into account to ensure that the color scheme is complete. Consequently, when the system grows, the color spectrum expands substantially [13].

The colour scheme and materials used in color quality is heavily influenced by the materials and its texture. Materials such as pigments, dyes, and inks are thus essential to color design [14]. The relevance of color matching in the design of visual media communication may be seen from this example. “Because of the rise of digital media, visual communication design has also experienced significant transformations [15].” The features of the system must be examined in order to enhance its execution. In terms of guiding features, this is one of the most important aspects of digital media. An unintentional but deliberate pursuit of a scientific and complete understanding of visual qualities is part of the visual communication design process [16]. When people are reading, the internal connections are more visible. When people use graphic representations in our communications, people can convey our everyday routines and the rules of nature more clearly. As a result, visual communication design plays a significant part in strategic planning [17]. Visible outcomes can only be seen if the strategic implementation strategy is strengthened.

Interaction is the next step. Both must be taken into account if visual design is to be continually improved. The interactions and limits of traditional optical systems are rather significant [18]. Because of this significant restriction, there has been progress in the link between visual design and the media, and this has helped to enhance visual design while simultaneously increasing the influence of the media on it. Visual communication design is driven by humanitarianism from a human perspective [19]. To put it another way, developing visual communication skills serves not only the spiritual but also the physical, material, and spiritual requirements of individuals. It is essential that every visual design adheres to the humanitarian principle in order to maximize its worth [20]. To sum it up, diversity is primarily the means through which designers get knowledge, with integration serving as a complement. It is becoming more popular and ideal as the designer's creative visual communication design evolves [21]. Ultimately, the goal of the merger is to bring together academic expertise in visual communication design in order to improve visual communication design's overall integrity and layout [22]. Visual communication designers know that color is the most effective tool for grabbing a viewer's attention out of all the elements at their disposal. Colorful LED tubes are used to create a magical real environment by the designer [23]. They feel like they are in the Milky Way with the development of the neon lights that flicker in the sky. The whole subway atmosphere is made more visually appealing with the employment of a powerful composition color design [24].

AI is the English term for intelligence. New scientific theories, methods, technologies, and systems are continually being developed in research and simulation. For visual media communication design, AI technology may offer a more effective presenting platform, enhance audience delight, and assist designers in completing more convenient colors using AI technology and simulation trials [25]. The use of artificial intelligence (AI) in visual media communication design may lead to improved image perception. Machine vision and picture recognition technologies, on the other hand, may assist in broadening the scope of the design concept for visual media communication [26]. In addition, the audience is better equipped to absorb and make sense of what is being spoken. These branches of study may be considered to have transcendental qualities. The link between cognitive science and artificial intelligence is the relationship between theory and practice. From a thinking perspective, artificial intelligence is not restricted to logical reasoning. People need to do research on visual thinking and exciting thinking in order to advance artificial intelligence [27]. Visual communication design relies heavily on people's preferences and understanding of color. An efficient visual system that helps users to identify similarities and differences between components is best created by designers by employing colors deliberately and strategically rather than using an excessive number of colors. It is also necessary to take into account the color's saturation and the space filled by colors close to it [28]. The user's visual senses will be overwhelmed if the interface is excessively vivid and employs too many colors. When it comes to choosing colors for an interface, the demands of both the brand and the interface might clash. It is because the connotations of various colors vary from culture to culture [29]. As a result, before deciding on colors for the intended audience, double-check the connotations of each individual hue and color combination. There is no existing study performed on the topic of APP interface design using AI. Hence, this study focused on applying visual communication in APP interface design using deep learning techniques.

## 3. Materials and Methods

In this work, a new enhanced deep learning-based automated historical image colorization in wireless network-enabled visual communication (EDL-AHIC) technique has been developed for automatically colorizing the grayscale cultural images. The proposed EDL-AHIC technique involves the design of convolutional neural network (CNN) with the ECN model. Primarily, the EDL-AHIC technique extracts the low-level features from the image which are then employed to determine mid-level features. Secondly, the ECN model is applied to derive global features. Finally, the decoding unit receives the outcome from the fusion layer, which acts as the “colorization network” that provides the final chrominance map.

### 3.1. Preprocessing

Firstly, an arbitrary set of RGN and grayscale images is used for training and testing datasets. The images with different aspect ratios and poor resolution are discarded from the dataset. Next, the images are cropped and resized into 256 ^∗^ 256 pixels. Afterward, 256 ^∗^ 256 ^∗^ 3 images are transformed into CIE *L*^*∗*^*a*^*∗*^*b*^*∗*^ color model since the presented approach transforms the RBG image into respective color layers, namely, two chromas and luminance (L that contains image features) components.

### 3.2. ECN-Based Global Feature Extraction

The CNN model involves a sequence of layers. An input map was moved with the individual's layer still achieving the resultant map. Detailed individual layers are provided to illustrate the computation equation. Assume that *X* ∈ *R*^*h*×*w*×*c*^(*h*: height, *w*: width, and *c*: channel) is an RGB image. All the layers get *X* and a group of parameters *W* as input and output a novel image *y* ∈ *R*^*h*′×*w*′×*c*′^, i.e., *y*=*f*(*X*, *W*). In the ECN algorithm, the divided pixel set of images is labeled as a group of nerve cells equivalent to capsules. The pixel vector was utilized as activation vector between active capsules, and it can be particular classes like healthy/tumor to a segmentation image dependent upon the pixel vector which signifies the entire lengths. The capsule routing from a layer was carried out through the multiplication of capsule outcome and the coupling coefficient (CC) (weighted matrix). The values of CC were defined as the resistance of parent capsule to route. The minimum level tumor analysis was determined as maximum level capsule activation with top‐down feedback process technique that is named as “routing‐by‐agreement.” Assuming *Y*_*i*_∈ [healthy, tumor] as resultant capsule *i*, *we*_*ij*_ represents the weighted matrix:

(1) $$\begin{array}{c} {\hat{y}}_{\left(ji\right)}=we_{ij}y_{i}, \end{array}$$

where ${\hat{y}}_{\left(ji\right)}$ determines the recognition vector which analysis the resultant parent capsule *j* utilizing capsule *i* and pixel ranges are utilized to estimate the weighted amount as in equation (1). The amount to the weighted was enhanced only if the value is reduced or pixel contains possible to positive class. The softmax function was utilized by means of the previous layer capsule and potential parent capsule as coefficient was encryption *c*_*ij*_ whereas an initial logits *b*_*ij*_ illustrates the log preceding possibility of routing capsule value *i* from the preceding layer for capsule value *j* from the subsequent layers.  Figure 1 depicts the structure of CapsNet.

Usually, the “routing‐by‐agreement” approach was executed as logits of capsules from each layer as follows:

(2) $$\begin{array}{c} c_{ij}=\frac{e^{b_{ij}}}{\sum_{i}e^{b_{ij}}}. \end{array}$$

The preceding layer illustrates a vital component from the computation of input of the parent capsule *j* that is gained as

(3) $$\begin{array}{c} s_{j}=\sum_{i}c_{ij}{\hat{y}}_{\left(j|i\right)}. \end{array}$$

The compression value of pixel vectors is introduced from the range of zero and one, utilizing a nonlinear function named squashing. The calculation function was expressed as

(4) $$\begin{array}{c} va_{j}=\frac{{\left\|s_{j}\right\|}^{2}}{1+{\left\|s_{j}\right\|}^{2}}\times \frac{s_{j}}{\varepsilon +{\left\|s_{j}\right\|}^{2}}, \end{array}$$

where *ε*=10^−7^.

Also, the following layer capsule was obtained:

(5) $$\begin{array}{c} a_{ij}=va_{j}\times {\hat{y}}_{\left(ji\right)}.\; \end{array}$$

The total capsule classifier that is considered as separate margin loss (Loss_*k*_) from all category capsules *k* to capsule network dependent upon the loss is as follows:

(6) $$\begin{array}{c} {\text{Loss}}_{k}=T_{k}\;\max\;{\left(0,m^{+}-\left\|va_{k}\right\|\right)}^{2}+\lambda \left(1-T_{k}\right)\max{\left(0,\left\|va_{k}\right\|-m^{-}\right)}^{2}, \end{array}$$

where *T*_*k*_ implies the instantiation occurrence from category capsules *k* and *λ*, *m*^−^, and *m*^+^ refer to the hyperparameter supports. The trained ECN was introduced based on 600 iterations according to Adam optimization for better hyperparameter with the rate of learning the amount of layered capsules 1*e* − 5.

### 3.3. Optimization and Learning Process

An objective function is for finding optimum value to model parameters with minimized cost (or loss) function. In order to measure the model loss quantitatively, there are two various tries developed, one is MSE and other is PSNR (Peak signal to Noise Ratio). The MSE was computed amongst the evaluated pixel color from *a*^*∗*^*b*^*∗*^ space and its ground truth value. In order to image *P*, the MSE has been provided as

(7) $$\begin{array}{c} C\left(P,\beta \right)=\frac{1}{2HW}\;\sum_{k\in \left\{a,b\right\}}\sum_{i=1}^{H}\sum_{j=1}^{W}{\left(P_{k_{i,j}}-{\tilde{P}}_{k_{i,j}}\right)}^{2}, \end{array}$$

where *C*(*P*, *β*) refers to the loss functions, *β* denotes the model parameter, and *P*_*k*_*i*,*j*__ and ${\tilde{P}}_{k_{i,j}}$ represent the *i*, *j*th pixel value of *k*th elements of forecasted and ground truth image correspondingly. To all the iterations, the loss was BP for updating the model parameter *β* utilizing the Adam optimization with global rate of learning *η*=0.001. The PSNR is another main quality assessment metric presented for measuring the quality of forecasted color images. The PSNR computes the PSNR amongst colorized images and equivalent ground truth images. The PSNR (in dB) was formulated as

(8) $$\begin{array}{c} \text{PSNR}=10\log_{10}\left(\frac{\text{peak }{\text{val}}^{2}}{\text{MSE}}\right)\\ =20\log_{10}\left(\text{peak val}\right)-10\log_{10}\left(\text{MSE}\right), \end{array}$$

where peak val (peak value) is the maximal value to pixel intensity of images. The peak value may be in the range of 255 to 8bits pixel representation.

## 4. Results and Discussion

The experimental result analysis of the EDL-AHIC technique with recent approaches is carried out in this section. The results are inspected for MSE, RMSE, accuracy, and training time.  Figure 2 illustrates the sample images of input black and white image.  Figure 3 demonstrates the sample of output colorized image.

Table 1 offers a detailed comparative study of the EDL-AHIC technique with recent methods.

Figure 4 depicts the comparative MSE examination of the EDL-AHIC technique with existing techniques. The figure reported that CNN-Inception (100) has shown poor performance with the MSE of 1911.000. Likewise, the CNN-Inception (200) model has tried to exhibit slightly enhanced outcomes with the MSE of 608.000. But the EDL-AHIC technique has surpassed the other two models with the MSE of 502.000.

Figure 5 portrays the comparative RMSE study of EDL-AHIC system with current methodologies. CNN-Inception (100) has revealed poor performance with the RMSE of 43.715. Likewise, the CNN-Inception (200) system has attempted to show slightly improved results with the RMSE of 24.658. However, the EDL-AHIC approach has exceeded the other two methods with the RMSE of 22.405.

Figure 6 represents the comparative study of the EDL-AHIC algorithm with current models. CNN-Inception (100) has shown poor performance with the accuracy of 0.671. Likewise, the CNN-Inception (200) method has attempted to display slightly improved results with the accuracy of 0.752.

However, the EDL-AHIC approach has exceeded the other two algorithms with the accuracy of 0.796.

Figure 7 demonstrates the comparative training time (TT) study of the EDL-AHIC system with present methods. CNN-Inception (100) has shown poor performances with the TT of 156.600 min. Likewise, the CNN-Inception (200) method has attempted to display slightly improved outcomes with the TT of 375.000 min. However, the EDL-AHIC approach has exceeded the other two approaches with the TT of 311.230 min.

Therefore, the EDL-AHIC technique can automatically colorize the images compared to existing techniques.

## 5. Conclusions

It is possible to educate visual communication designs using linguistics or semiotics, making it an innovative and scientific field. When storytelling techniques are used in visual communication, a designer's creativity and the audience's visual memory are enhanced. In addition, preserving historical images and other forms of cultural heritage is essential if we are to maintain our rich cultural diversity. Colorization of grayscale photos has been made possible by advances in deep learning (DL) and computer vision (CV) techniques in recent years. EDL-AHIC is a new technology for wireless visual communication based on enhanced deep learning-based automatic historical image colorization (EDL-AHIC). Effective colorization of grayscale photos will be achieved with EDL-AHIC. Local and global characteristics can both be extracted using the EDL-AHIC method that we have demonstrated. The expanded capsule network (ECN) model is used to extract global features. Finally, the output image's chrominance component is determined using the fusion layer and decoding unit. To ensure that the EDL-AHIC technique is improved, a complete experimental validation process is carried out. The EDL-AHIC methodology was found to be superior to other recent technologies in a comparison study.

## Figures and Tables

**Figure 1:** Framework of CapsNet.

**Figure 2:** Input black and white image.

**Figure 3:** Output colorized image.

**Figure 4:** MSE analysis of EDL-AHIC technique with recent methods.

**Figure 5:** RMSE analysis of EDL-AHIC technique with recent methods.

**Figure 6:** Accuracy analysis of EDL-AHIC technique with recent methods.

**Figure 7:** Training time analysis of EDL-AHIC technique with recent methods.

**Table 1:** Comparative analysis of EDL-AHIC technique with recent approaches.

Methods	MSE	RMSE	Accuracy	Training time (min)
CNN-Inception (100)	1911.000	43.715	0.671	156.600
CNN-Inception (200)	608.000	24.658	0.752	375.000
EDL-AHIC	502.000	22.405	0.796	311.230

## Data Availability

The data used to support the findings of this study are available from the corresponding author upon request.
